This article has been retracted.

# Long non-coding RNA H19 aggravates keloid progression by upregulating SMAD family member 5 expression via miR-196b-5p

**DOI:** 10.1080/21655979.2021.2019868

**Published:** 2022-01-03

**Authors:** Zhichao Li, Cheng Gong, Huiming Wei

**Affiliations:** a Department of Hand and Foot Microsurgery, Hanyang Hospital Affiliated to Wuhan University of Science and Technology, Wuhan, Hubei, China; b Department of Dermatological, Huazhong University of Science and Technology and Jiangbei Hospital, Wuhan, Hubei, China; c Department of Medical and Beauty, Huazhong University of Science and Technology and Jiangbei Hospital, Wuhan, Hubei, China

**Keywords:** lncRNA H19, miR-196b-5p, smad5, keloid

## Abstract

Accumulating evidence suggests that long non-coding RNAs (lncRNAs) participate in the formation and development of keloids, a benign tumor. In addition, lncRNA H19 has been shown to act on the biological processes of keloids. This study aimed to identify other important mechanisms of the effect of lncRNA H19 on keloid formation. The H19, miR-196b-5p, and SMAD family member 5 (SMAD5) expression levels were detected using quantitative reverse transcriptase polymerase chain reaction (qRT-PCR) and Western blotting. Subcellular localization of lncRNA H19 was detected using a nuclear–cytoplasmic separation assay. Cell viability and proliferation were measured using counting kit-8 and colony formation assays. Bax and Bcl-2 levels were examined using Western blot analysis. The interaction between H19 and miR-196b-5p or SMAD5 was verified using a dual-luciferase reporter assay. H19 and SMAD5 expression was upregulated in keloid tissue and fibroblasts, whereas miR-196b-5p expression was downregulated. Knockdown of H19, overexpression of miR-196b-5p, or knockdown of SMAD5 inhibited the viability and proliferation of keloid fibroblasts and promoted apoptosis. Overexpression of H19 or SMAD5 and knockdown of miR-196b-5p promoted viability and proliferation and inhibited apoptosis. miR-196b-5p was identified as a H19 sponge, and SMAD5 was identified as a miR-196b-5p target. The combination of lncRNA H19 and miR-196b-5p regulates SMAD5 expression and promotes keloid formation, thus providing a new direction for keloid treatment.

## Introduction

Keloid is a biological phenomenon in which the growth of the wound surface exceeds the boundary of the original injury during wound healing and is a benign skin tumor [1]. Pathologically, keloids manifest as abnormal collagen bundles and abnormal hyperplasia of capillaries. At the cellular level, it manifests an excessive proliferation of fibroblasts, inhibited apoptosis, and secretion of a large amount of extracellular matrix (ECM) [2,3]. Previous research has reported that keloids demonstrate a higher prevalence in certain races and alterations in gene expression favor a significant genetic contribution to keloid pathology, suggesting that the genetic basis is an important factor in the development of keloids [4].

Accumulating evidence suggests that the pathogenesis of keloids is related to the functional activity of various genes and cytokines [5]. Long non-coding RNAs (lncRNAs) have been shown to participate in various biological processes such as cell proliferation and apoptosis [6]. Recently, various lncRNAs have been shown to be involved in keloid disease progression. The lncRNA HOXA11-AS expression was upregulated significantly in keloid tissues or fibroblasts, and the overexpression of HOXA11-AS inhibited the apoptosis of keloid cells and promoted angiogenesis induced by fibroblasts [7]. The lncRNA CACNA1G-AS1 expression is upregulated in keloid fibroblasts, promotes cell proliferation and invasion, and inhibits cell apoptosis [8]. lncRNA H19 has been shown to be upregulated in many malignant and benign tumors. Furthermore, H19 plays an important role in cell proliferation, migration, and invasion; ECM deposition; and vascular endothelial growth factor secretion in keloid formation [9–11].

lncRNAs act as microRNA (miRNA) sponges, and miRNAs inhibit mRNA expression through mRNA cleavage and/or direct translation, thus regulating disease development and progression after transcription [12]. Literature indicates that lncRNA H19 promotes fibroblast proliferation and metastasis by regulating the downstream miR-29a/COL1A1 axis [9]. lncRNA NEAT1 silencing inhibits malignant proliferation and ECM expression in keloid fibroblasts by modifying miR-196b-5p and fibroblast growth factor 2 (FGF2) expression [13]. The down regulation of LINC01116 expression regulates the miR-203/SMAD5 axis to inhibit keloid formation [14]. However, the mechanisms by which the H19/miR-196b-5p/SMAD5 axis modulates keloid formation has not yet been investigated.

The effects of H19, miR-196b-5p, and SMAD5 on the proliferation and apoptosis of keloid fibroblasts were investigated. We hypothesized that the potential regulatory networks of H19/miR-196b-5p/SMAD5 play a crucial role in keloid progression. This study aimed to explore a new mechanism for understanding the pathogenesis of keloid formation.

## Materials and methods

### Research object

Keloid and normal skin tissues were obtained from 17 keloid patients who underwent surgical resection in our hospital. None of the study participants received keloid treatment prior to the surgery. All procedures in this study were approved by the ethics committee of our hospital. Each participant signed a written informed consent form prior to surgery.

### Isolation and culture of primary fibroblast

Keloid fibroblasts and normal fibroblasts were isolated from keloid tissue and matched normal skin tissue. The freshly excised tissue was disinfected with alcohol and cut into 2 mm^3^ pieces. Adipose and connective tissues were removed and washed with PBS to remove blood stains. The tissue mass was incubated for 4 h at 37°C with 2.5 mg/mL dispase II (Sigma Aldrich, USA) solution and then incubated in DMEM (Invitrogen, USA) supplemented with 10% fetal bovine serum at 37°C and 5% CO_2_. Changes in cell morphology and color in the culture medium were observed daily. The third generation of cells was used in the follow-up experiments [15].

## Nucleocytoplasmic separation assay

The PARIS Kit (Thermo Fisher, USA) was used to separate nuclear and cytoplasmic fractions from keloid fibroblasts. After digestion, the cells were resuspended in the medium for a further 15 min and then homogenized. The cells were centrifuged for 15 min at 4°C for 400 ×* g*, and the cytoplasm was isolated from the supernatant. Using PBS, nuclear isolation buffer, and 0.3 mL RNase-free H_2_O, the precipitate was suspended in a centrifuge tube and incubated on ice for 20 min. The granules were then centrifuged to obtain the desired nuclear fragments. Using glyceraldehyde-3-phosphate dehydrogenase (GAPDH) as the cytoplasmic control and 18S as the nuclear control, the H19 expression was detected using quantitative reverse transcriptase polymerase chain reaction (qRT-PCR) in the cytoplasm or nucleus of keloid fibroblasts [16].

### Cell transfection

Small interfering RNA targeting H19 gene knock-out (50 nM; H19-siRNA-1, H19-siRNA-2, and H19-siRNA-3) and H19 overexpression plasmid (100 nM; pcDNA-H19) were assembled at Genepharma (China). Small interfering RNA targeting the SMAD5 gene knock-out (50 nM; si-SMAD5) and SMAD5 overexpression plasmid (100 nM; pcDNA-SMAD5) were provided by RiboBio (China). miR-196b-5p mimic (50 nM) and miR-196b-5p inhibitor (100 nM) were provided by Switch Gear (USA). In this study, Lipofectamine 3000 (Invitrogen) was used for transfection.

### qRT-PCR

For quantitative mRNA analysis, an RNeasy Plus Mini Kit (Qiagen, Hilden, Germany) was used to extract total RNA from skin tissues and fibroblasts. Reverse transcription of RNA into cDNA was performed using the PrimeScript reagent Kit (Takara). The cDNA was diluted, and qRT-PCR was performed on an ABI 7300 system (Thermo Fisher) using the SYBR Green Master Mix (Vazyme, China). The expression of H19 and SMAD5 was detected using qRT-PCR and normalized to that of GAPDH.

For quantitative miRNA analysis, total RNA was extracted using the miRNeasy Mini kit (Qiagen). RNA was reverse-transcribed into mature miRNA using the Bulge LoopTM miRNA qRT-PCR Starter Kit (Ribibio, China). The expression of miR-196b-5p was normalized to that of the small nuclear RNA 6 (U6). Gene expression was calculated using the 2^−ΔΔCt^ method [17]. The sequences of primers used in the study are listed in Table 1.

**Table 1.** PCR The sequences of the primers in this study

Primer	Sequences
**lncRNA-H19**	Forward: 5’-CTGGGCAACGGAGGTGTA-3’
	Reverse: 5’-CTGGGAGGGTGTCTGCTTC-3’
**SMAD5**	Forward: 5’-TTTCGCTAGCCAACTTTT-3’
	Reverse: 5’-TATCTGTTTTCAATGTAAGCTC-3’
**miR-196b-5p**	Forward: 5’-ATCCTTCCTAGTCCAGCCTGAG-3’
	Reverse: 5’-ACCTGGCGGCACTCCTTA-3’
**GAPDH**	Forward: 5’-AGGTCGGTGAACGGATTTG-3’
	Reverse: 5’-GGGGTCGTTGATGGCAACA-3’
**U6**	Forward: 5’-CTCGCTTCGGCAGCACATATACT-3’
	Reverse: 5’-ACGCTTCACGAATTTGCGTGTC-3’

### Luciferase activity assay

The partial length of H19 wild-type (H19-WT), H19 mutant (H19-MUT), SMAD5 wild-type (SMAD5-WT), and SMAD5 mutant (MUT1, MUT2, and Co-MUT) were synthesized and inserted into the pGL3 luciferase vector (Promega, USA). The 3’-UTRs of H19 and SMAD5 mutant sequences were synthesized at Sangon Biotech (China). Keloid fibroblasts were inoculated into 96-well plates at a confluence of 70%. The luciferase reporter gene plasmid, miR-196b-5p mimic, miR-196b-5p inhibitor, or miR-NC were transfected into cells 16 h after inoculation. Luciferase activity was detected using the firefly luciferase assay kit (Promega) [18].

### Cell counting kit (CCK)-8 assay

Keloid fibroblasts transfected for 48 h (5 × 10^3^ cells) were seeded into 96-well plates, cultured for 0, 24, 48, or 72 h in an incubator, and further analyzed using the CCK-8 kit (Beyotime, China). The supernatant of the cultured cells was removed and 100 μL of complete medium containing 10 μL of CCK-8 solution was added to each well for 1 h. The absorbance at 450 nm was recorded using a microplate analyzer (BioTek, USA) [19].

### Colony formation assay

In this experiment, 1000 keloid fibroblasts transfected for 24 h were inoculated into 6-well plate and cultured in an incubator for 2 weeks. The colonies were fixed with 10% methanol at 25°C for 15 min and stained with 0.1% crystal violet for 20 min; subsequently, more than 50 cell colonies were counted under the microscope [20].

### Western blot analysis

Western blotting was performed as described previously [21]. Total protein lysates were obtained using radioimmunoprecipitation assay buffer containing protease inhibitors (Sigma Aldrich). Protein concentration in the lysates was determined using the bicinchoninic acid method (Sigma Aldrich). Quantitative proteins were transferred to polyvinylidene fluoride (PVDF) membranes after sodium dodecyl sulfate polyacrylamide gel electrophoresis (SDS-PAGE). Thereafter, 5% skimmed milk powder dissolved in PBS–0.2% Tween-20 (PBST) buffer was used to seal the PVDF membrane for 2 h at 25°C, and the membrane was incubated overnight with antibodies against SMAD5 (ab40771; 1:2000), Bax (ab32503; 1:1000), Bcl-2 (ab32124; 1:1000), and GAPDH (ab8245; 1:2000; all from Abcam, UK) at 4°C. Subsequently, horseradish peroxidase-labeled secondary antibodies were added, followed by incubation at room temperature for 1 h. PBST post-wash enhanced chemiluminescence (Pierce, USA) was used to detect the protein bands, and the signal strength was quantitatively measured using the ImageJ software (NIH, USA).

### Statistical analyses

All data obtained in this study are presented as the mean ± standard deviation. The Student’s *t*-test was performed to compare the data between two groups. One-way analysis of variance was performed to test the data among multiple groups. Pearson correlation analysis was used to study the correlation between H19 and miR-196b-5p expression in keloid tissue, and the correlation between the two variables was described and analyzed using correlation coefficients and scatter plots. All statistical analyses were performed using GraphPad Prism 6.0 (GraphPad Software, USA). Statistical significance was set at p < 0.05.

## Results

This study aimed to explore the downstream mechanisms by which H19 affects keloids. We conducted a series of in vitro experiments and found that H19 promoted the viability and proliferation of keloid fibroblasts and inhibited apoptosis by regulating the miR-196b-5p/SMAD5 axis. Therefore, our data for the first investigation of the functional and clinical expression changes of H19/miR-196b-5p/SMAD5 in keloids provide new insights into the pathogenesis of keloids.

### miR-196b-5p expression was potentially downregulated by H19 in keloids

H19 has been reported to aggravate keloid progression in several studies [9,11]. We also found that the SMAD family has been frequently reported to be involved in keloid progression. In particular, SMAD5 was significantly upregulated in keloids and promoted keloid formation and development [14,22]. To identify a potential link between H19 and SMAD5, we interrogated the starBase database to predict the targets of H19 and SMAD5. A total of 51 common miRNAs were identified (Figure 1(a)). We found relevant research regarding the 51 miRNAs. In addition, we found that miR-196b-5p was reported to be a significant suppressor in keloids [13]. In addition, miR-196b-5p was predicted to be the target of H19, with the second most significant miRNA target according to the number of supported AGO CLIP-seq experiments using the starBase algorithm. In our experiments, we detected H19 expression in the keloid tissues we collected. H19 was found to be significantly overexpressed in keloids (Figure 1(b)). We also found that miR-196b-5p was downregulated in keloids (Figure 1(c)). The expression of H19 and miR-196b-5p in keloid tissues was negatively correlated (Figure 1(d)). Moreover, cell fractionation qRT-PCR experiments showed that H19 was primarily located in the cytoplasm (Figure 1(e)).

**H19 targeted miR-196b-5p in keloids**

**Figure1.** **miR-196b-5p is downregulated and potentially regulated by H19 in keloid**. A. The target miRNAs that potentially link H19 and SMAD5 mRNA. The target miRNAs were predicted using starbase algorithm. B. The expression of H19 in keloid tissues. C. The expression of miR-196b-5p in keloid. **P < 0.01compared with normal fibroblasts. D. The relationship between H19 expression and miR-196b-5p expression in keloid tissues. E. The localization of H19 in cell.

The above data showed a negative correlation between H19 and miR-196b-5p in keloids. Thereafter, we determined the relationship between H19 and miR-196b-5p expression. Analysis using starBase revealed the presence of targeted sites for H19 binding to miR-196b-5p (Figure 2(a)). To determine the relationship between H19 and miR-196b-5p, a dual-luciferase reporter assay was performed. Luciferase activity was found to decrease after co-transfection of wild-type H19 with miR-196b-5p mimic and increased after co-transfection of wild-type H19 with miR-196b-5p inhibitor; however, it was not affected by co-transfection of mutant H19 with miR-196b-5p mimic (Figure 2(b)), revealing that miR-196b-5p bound to H19. Further investigation of H19 expression in keloid fibroblasts showed a 6-fold increase in H19 levels after transfection with pcDNA-H19 and a decrease of 80%, 70%, and 60% after transfection with the three H19 knockdown plasmids (Figure 2(c)). H19-siRNA-1 was used in subsequent experiments. miR-196b-5p expression was regulated, and it was shown that the level of miR-196b-5p increased three times after overexpression of miR-196b-5p and decreased by 70% after expression of miR-196b-5p was downregulated (Figure 2(d)).

**H19 promoted the proliferation of keloid cells via miR-196b-5p**

**Figure 2.** **miR-196b-5p H19 targets miR-196b-5p in keloids**. A. The seed regions of miR-196b-5p, the seed-recognizing sites in the H19 are shown. B. Luciferase activity of wild-type H19 and mutant H19 constructs in keloid fibroblast after transfection with miR-196b-5p mimic or miR-196b-5p inhibitor. **P < 0.01compared with miR-NC. C. Keloid fibroblast were transfected with pcDNA-H19, H19-siRNA-1, H19-siRNA-2 and H19-siRNA-3. The expression of H19 was detected by QRT-PCR after transfection. *P < 0.05, **P < 0.01compared with NC. D. Keloid fibroblast were transfected with miR-196b-5p mimic and miR-196b-5p inhibitor. The expression of miR-196b-5p was detected by QRT-PCR after transfection. **P < 0.01compared with miR-NC.

Thereafter, the proliferation and apoptosis of keloid fibroblasts affected by H19 and miR-196b-5p were studied. CCK-8 assay showed that cell viability increased after overexpression of H19 or knockdown of miR-196b-5p and decreased after interference with H19 or upregulation of miR-196b-5p expression (Figure 3(a)). Similarly, cell proliferation was further measured using a cell colony formation assay. The colony number of cells transfected with pcDNA-H19 or miR-196b-5p inhibitor was approximately 2.3 times and 2 times more than that of the NC group, respectively. The colony number of cells transfected with H19-siRNA or miR-196b-5p mimic was approximately 70% and 60% of the NC group, respectively (Figure 3(b)). Furthermore, Bax and Bcl-2 protein expression was detected using Western blotting to verify the changes in apoptosis. Compared to that in the NC group, Bax protein content decreased and Bcl-2 increased after transfection with pcDNA-H19 or miR-196b-5p inhibitor, whereas Bax protein content increased and Bcl-2 decreased after transfection with H19-siRNA or miR-196b-5p mimic (Figure 3(c)).

**Figure 3.** **H19 promotes the proliferation and inhibited apoptosis of keloid cells through miR-196b-5p**. A. CCK-8 assay was analyzed cell viability in keloid fibroblast transfected with pcDNA-H19, H19-siRNA, miR-196b-5p mimic or miR-196b-5p inhibitor. B. Colony-forming assay was used to assess the effect of H19 and miR-196b-5p on cells proliferation in keloid fibroblast. C. Western blot analysis was performed to measure the expression of Bax and Bcl-2, GAPDH was used as a loading control. **P < 0.01compared with NC.

### SMAD5 was the target gene of miR-196b-5p

Analysis using starBase revealed two targeting sites for SMAD5 and miR-196b-5p (Figure 4(a)). The wild-type reporter vector and mutated reporter vector of SMAD5 were synthesized. The analysis showed that the luciferase activity decreased by 60% after co-transfection of WT and miR-196b-5p mimics, by 40% after co-transfection of MUT1 and miR-196b-5p mimics, by 30% after co-transfection of MUT2 and miR-196b-5p mimics, and insignificantly after transfection of co-MUT and miR-196b-5p mimics (Figure 4(b)). In addition, luciferase activity increased after co-transfection of WT, MUT1, or MUT2 with miR-196b-5p inhibitor, whereas there was no significant change in luciferase activity after co-MUT and miR-196b-5p inhibitor transfection (Figure 4(b)). It was revealed that miR-196b-5p targeted SMAD5. qRT-PCR showed that SMAD5 mRNA expression in keloid tissues increased 2.5-fold (Figure 4(c)). Western blotting showed that SMAD5 protein levels in keloid tissue were also increased (Figure 4(d)). Pearson analysis indicated a negative correlation between SMAD5 and miR-196b-5p in keloid tissue (Figure 4(e)).

**Figure 4.** **SMAD5 is the target gene of miR-196b-5p**. A. A wild/mutant type SMAD5 3’-UTR reporter (or control construct) and miR-196b-5p plasmid (or control plasmid) were transduced into keloid fibroblast. B. The dual-luciferase reporter gene assay was performed to identify the interaction between SMAD5 and miR-196b-5p. Luciferase activities were calculated as the ratio of firefly/renilla activities. **P < 0.01compared with miR-NC. C. QRT-PCR was used to determine the expression of SMAD5 mRNA in normal skin tissues and keloid tissues. D. Western blot was used to determine the expression of SMAD5 protein in normal skin tissues and keloid tissues. **P < 0.01compared with normal tissue. E. Pearson analysis was used to analyze the association between miR-196b-5p and SMAD5 expression.

### SMAD5 expression was increased in keloid fibroblast

To determine the expression of SMAD5 at the cellular level, qRT-PCR was first used, which showed that the SMAD5 mRNA expression level in keloid fibroblasts was approximately 3.3 times higher than that in normal fibroblasts (Figure 5(a)). Second, Western blotting showed a 1.6-fold increase in SMAD5 protein expression in keloid fibroblasts (Figure 5(b)). Further detection of SMAD5 in keloid fibroblasts revealed a 1.3-fold or 1.2-fold increase in SMAD5 protein levels in pcDNA-H19 or miR-196b-5p inhibitor groups and a 70% or 30% decrease in SMAD5 protein levels in H19-siRNA or miR-196b-5p mimic groups (Figure 5(c)).

**Figure 5.** **SMAD5 expression is increased in keloid cells**. A. SMAD5 mRNA in normal fibroblasts and keloid fibroblast. B. SMAD5 protein in normal fibroblasts and keloid fibroblast. **P < 0.01compared with normal fibroblasts. C. Western blot analysis was performed to measure the expression of SMAD5 in H19/miR-196b-5p upregulated/downregulated groups. *P < 0.05, **P < 0.01compared with NC.

### miR-196b-5p was involved in the proliferation and apoptosis of keloid fibroblast via SMAD5

Thereafter, the expression level of SMAD5 was regulated, and Western blotting revealed that the SMAD5 expression protein was upregulated by approximately 1.3 times after transfection of pcDNA-SMAD5 and downregulated by more than 50% after transfection with si-SMAD5 (Figure 6(a)). The CCK-8 assay showed a 1.5-fold increase in cell viability after overexpression of SMAD5 and a 60% decrease after downregulation of SMAD5 expression (Figure 6(b)). Moreover, si-SMAD5 and pcDNA-SMAD5 reversed the effect of miR-196b-5p inhibitor and miR-196b-5p mimic on cell viability, respectively (Figure 6(b)). Colony formation assay showed that SMAD5 knockdown increased colony number and reversed the proliferative effect of miR-196b-5p inhibitor, whereas overexpression of SMAD5 reduced colony number and partially eliminated the inhibitory effect of the miR-196b-5p mimic (Figure 6(c)). Furthermore, Western blot analysis showed that in contrast to the miR-NC group, the protein content of Bax decreased and Bcl-2 increased in the miR-NC + pcDNA-SMAD5 group, whereas the opposite trend was observed in the miR-NC + si-SMAD5 group (Figure 6(d)). Moreover, silencing or overexpression of SMAD5 reversed the effects of interference or upregulation of miR-196b-5p on Bax and Bcl-2 protein levels (Figure 6(d)).

**Figure 6.** **miR-196b-5p is involved in the proliferation and apoptosis of keloid fibroblast through SMAD5**. A. Western blot analysis was performed to measure the expression of SMAD5 in SMAD5 upregulated and downregulated groups. **P < 0.01compared with NC. B. CCK-8 assay reveals the effect of SMAD5 on cell viability in keloid fibroblast with or without upregulation of miR-196b-5p. C. Colony-forming assay was used to assess the effect of SMAD5 and miR-196b-5p on cells proliferation in keloid fibroblast. D. Western blot analysis was performed to measure the expression of Bax and Bcl-2, GAPDH was used as a loading control. **P < 0.01compared with miR-NC.

## Discussion

Keloid, a benign skin tumor, is not treated effectively [23]. Fibroblasts are known as the key effector cells for keloid formation, and dysfunctions such as abnormal cell proliferation, metastasis, and overproduction of ECM have been identified in keloid formation [24]. Therefore, finding a molecular target that may prevent fibroblast dysfunction may be an effective way to treat keloids.

This study found that H19 was overexpressed in keloid tissues and fibroblasts. A previous study suggested that the abundance of H19 in keloid tissue and fibroblasts was significantly increased, and its downregulation inhibited cell proliferation [11]. Xu et al. [10] have shown that downregulation of H19 expression inhibits the aberrant proliferation and ECM deposition of keloid fibroblasts and promotes apoptosis. Wang et al. [9] collected 80 keloid tissues and isolated fibroblasts and found that PCDNA3.1-H19 could enhance the viability, proliferation, migration, and invasion of fibroblasts, whereas silencing H19 significantly inhibited the metastasis and proliferation of fibroblasts. Our data are consistent with those reported in the literature. Based on previous studies, we found that H19 knockdown inhibited the viability, proliferation, and Bcl-2 protein expression levels of keloid fibroblasts and promoted the expression of Bax protein through biological function analysis. Furthermore, overexpression of H19 has been shown to have an opposite effect as that of H19 knockdown. In addition, nuclear–cytoplasmic separation experiments showed that H19 was mainly expressed in the cytoplasm, suggesting that H19 regulates keloid development by acting in the cytoplasm of keloid fibroblasts, thereby affecting the biological processes.

Based on the above studies, starBase, an online tool, was used to analyze the miRNAs that H19 might target, and dual-luciferase assay revealed that miR-196b-5p combined with H19, and its expression was downregulated in keloid tissue and keloid fibroblasts. Accumulating evidence has shown that miR-196b-5p overexpression inhibits cell migration and viability and production of type I collagen, α-smooth muscle actin, and fibronectin of keloid fibroblasts [13]. On this basis, we found that miR-196b-5p knockdown promoted keloid fibroblast viability, plate clone number, and Bcl-2 protein level while inhibiting Bax protein level. These data indicate that miR-196b-5p inhibits keloid formation.

Drosophila mothers against decapentaplegic (SMAD) family member 5 (SMAD5) is a well-known transcription factor that plays a crucial role in cell proliferation, differentiation, migration, and apoptosis [25]. In this study, SMAD5 was found to be overexpressed in keloids. As a target of miR-196b-5p, SMAD5 promotes keloid fibroblast proliferation and inhibits apoptosis. Moreover, previous studies by Yuan et al. [14] and Jin et al. [22] found that SMAD5 knockdown inhibits keloid fibroblast proliferation and metastasis and production of ECM. It has been suggested that SMAD5 plays a role in promoting dysregulated proliferation in keloids.

Multiple lncRNA-miRNA-mRNA network mechanisms are involved in the occurrence and development of keloids [26,27]. H19/miR-196b-5p/SMAD5 is only one element of the regulatory network, and it is crucial to recognize the upstream enrichment of H19 and the downstream regulatory pathway of SMAD5. Concurrently, it is also important to explore the variation of H19/miR-196b-5p/SMAD5 on the ECM secretion of keloid fibroblasts. This will further deepen our understanding of the molecular mechanism of keloids.

## Conclusion

In conclusion, our study showed that H19 and SMAD5 levels were upregulated in keloid tissue and fibroblasts, promoting the proliferation and inhibiting apoptosis of keloid fibroblasts, whereas miR-196b-5p was downregulated and had an opposite effect to that of H19 and SMAD5. These data provide a new pathway for H19 regulation in the process of keloid formation and further validate the possibility of H19 as a potential therapeutic target for keloid patients.

## Data Availability

The datasets used and analyzed during the current study are available from the corresponding author on reasonable request.

## Highlights

1. Knockdown of H19, overexpression of miR-196b-5p, or knockdown of SMAD5 inhibited the viability and proliferation of keloid fibroblasts and promoted apoptosis.

2. Overexpression of H19 or SMAD5 and knockdown of miR-196b-5p promoted viability and proliferation and inhibited apoptosis of keloid fibroblasts.

3. miR-196b-5p was identified as a H19 sponge.

4. SMAD5 was identified as a miR-196b-5p target.
